# Protective effect of tanshinone IIA against cardiac hypertrophy in spontaneously hypertensive rats through inhibiting the Cys-C/Wnt signaling pathway

**DOI:** 10.18632/oncotarget.14328

**Published:** 2016-12-28

**Authors:** Jun Feng, Hua-Wen Chen, Li-Juan Pi, Jin Wang, Da-Qian Zhan

**Affiliations:** ^1^ Department of Emergency Medicine, Tongji Hospital, Huazhong University of Science and Technology, Wuhan 430030, Hubei, P.R. China

**Keywords:** tanshinone IIA, cardiac hypertrophy, Cys-C/Wnt signaling pathway, spontaneously hypertensive rats

## Abstract

The study aimed to investigate the protective effect of tanshinone IIA against cardiac hypertrophy in spontaneously hypertensive rats (SHRs) through the Cys-C/Wnt signaling pathway. Thirty SHRs were randomly divided into cardiac hypertrophy, low- and high-dose tanshinone IIA groups. Ten Wistar-Kyoto rats were selected as control group. The systolic blood pressure (SBP), heart weight (HW), left ventricular weight (LVW) and body weight (BW) of all rats were recorded. HE staining and qRT-PCR were applied to observe the morphology of myocardial tissue and mRNA expressions of COL1A1 and COL3A1. ELISA and Western blotting were used to measure the serum asymmetric dimethylarginine (ADMA), nitric oxide (NO) and cardiac troponin I (cTnI) levels, and the expressions of the Cys-C/Wnt signaling pathway-related proteins, eNOS and Nox4. Compared with the cardiac hypertrophy group, the SBP, HW/BW, LVW/BW, swelling degree of myocardial cells, COL1A1 and COL3A1 mRNA expressions, serum cTnI and ADMA levels, and the Cys-C/Wnt signaling pathway-related proteins and Nox4 expressions in the low- and high-dose tanshinone IIA groups were decreased, but the endothelial NO synthase (eNOS), phosphorylated eNOS (Ser1177) and NO expressions were increased. No significant difference was found between the low- and high-dose tanshinone IIA groups. Our study indicated a protective effect of tanshinone IIA against cardiac hypertrophy in SHRs through inhibiting the Cys-C/Wnt signaling pathway.

## INTRODUCTION

Hypertension (HTN), the third leading killer in the world and the most important risk factor for both cerebrovascular and cardiovascular diseases, is known as a chronic medical condition in which the blood pressure is constantly elevated in the arteries [1–3]. It is estimated that the incidence of HTN is approximately one third in young adults, 60% in those over 60 and 75% in people older than 70 years [4]. To the best of our knowledge, HTN can be divided into two categories clinically: primary HTN whose medical cause cannot be identified so far and secondary HTN which occurs as a result of other conditions affecting kidney, heart or artery disease [5]. Besides, one of the most important risk factors related to HTN is cardiac hypertrophy, a heart muscle thickening that causes the enlargement of ventricles, which is the primary reaction of the myocardium in response to mechanical overload or stress [6]. The Wnt signaling pathway plays a very important role in the development of cardiac hypertrophy [7]. Thus, the inhibition of Wnt signaling pathway can provide a new therapeutic strategy for cardiac hypertrophy [8].

Danshen, a widely used Chinese herbal medicine and an approved pharmacological compound, is obtained from the dried root or the rhizome of *Salvia miltiorrhiza Bge* [9]. Its extracts contain diterpene quinone and phenolic acid derivatives, including tanshinone (I, IIA and IIB), cryptotanshinone, isocryptotanshinone, miltirone, tanshinol (I and II) and salviol [10]. As is known so far, Danshen is used either alone or in combination with other herbal ingredients to prevent and manage many kinds of cardiovascular diseases, including myocardial infarction, HTN, stroke and angina pectoris, in China and other Asian countries [11, 12]. Tanshinone IIA, the most abundant diterpene quinone in Danshen, is clinically used in the treatment of cardiovascular and inflammatory diseases due to its minimal side effects [13]. Recently, tanshinone IIA was also demonstrated to have the abilities of inducing cell death and apoptosis in a variety of tumors, such as colon cancer, renal cell carcinoma, osteosarcoma and leukemia [14–17]. However, little is known about whether tanshinone IIA can inhibit cardiac hypertrophy in spontaneously hypertensive rats (SHRs). So, we aimed to investigate the mechanism by which tanshinone IIA inhibits cardiac hypertrophy in SHRs through the cystatin C (Cys-C)/Wnt signaling pathway.

## RESULTS

### Comparison of the SBP in the rats among the cardiac hypertrophy, low- and high-dose tanshinone IIA and control groups

As shown in Figure 1, before the experiment, the SBPs in the cardiac hypertrophy, low- and high-dose tanshinone IIA groups were 209.12 ± 9.74 mmHg, 204.45 ± 10.16 mmHg and 206.79 ± 8.69 mmHg, respectively. The SBPs in those three groups were obviously higher than that in the control group (all *P* < 0.05). Two and four weeks after the experiment, compared with the cardiac hypertrophy group, the low- and high-dose tanshinone IIA groups had decreased SBP, but the SBPs in the low- and high-dose tanshinone IIA groups were still higher than that in the control group (all *P* < 0.05). No significant difference was found between the low- and high-dose tanshinone IIA groups (all *P* > 0.05).

**Figure 1:** Comparison of SBP in the rats among the cardiac hypertrophy, low-dose tanshinone IIA, high-dose tanshinone IIA and control groups before the experiment, and at 2 and 4 weeks after the experiment Note: *, *P* < 0.05 compared with the control group; ^#^, *P* < 0.05 compared with the cardiac hypertrophy group; SBP, systolic blood pressure.

### Effect of tanshinone IIA on the cardiac hypertrophy indexes of SHRs

The cardiac hypertrophy indexes in the cardiac hypertrophy, low-dose tanshinone IIA, high-dose tanshinone IIA and control groups were shown in Table 1. The cardiac hypertrophy group had significantly higher HW/BW and LVW/BW when compared with the control group (all *P* < 0.05). Compared with the cardiac hypertrophy group, the low- and high-dose tanshinone IIA groups had significantly decreased HW/BW and LVW/BW (all *P* < 0.05), which were close to the normal levels (all *P* > 0.05).

**Table 1:** Comparisons of the cardiac hypertrophy indexes among the cardiac hypertrophy, low-dose tanshinone IIA, high-dose tanshinone IIA and control groups

Group	HW/BW	LVW/BW
Control group	3.26 ± 0.29	2.56 ± 0.24
Cardiac hypertrophy group	4.05 ± 0.33*	3.03 ± 0.19*
Low-dose tanshinone IIA group	3.57 ± 0.40^#^	2.77 ± 0.31^#^
High-dose tanshinone IIA group	3.44 ± 0.32^#^	2.64 ± 0.25^#^

Note: HW, heart weight; BW, body weight; LVW, left ventricular weight; *, *P* < 0.05 compared with the control group; ^#^, *P* < 0.05 compared with the cardiac hypertrophy group.

### Comparison of the morphological change in the myocardial tissue among the four groups

As shown in Figure 2, compared with the control group, the cardiac hypertrophy group had the swelling and sparsely arranged myocardial cells, increased single myocardial cell area, granular content, and karyopyknosis in some myocardial cells. These phenomena were improved partly in the low- and high-dose tanshinone IIA groups. Compared with the cardiac hypertrophy group, the swelling degree of myocardial cells was down-regulated and the single myocardial cell area decreased in the low- and high-dose tanshinone IIA groups, but there was no significant difference between the low- and high-dose tanshinone IIA groups (*P* > 0.05).

**Figure 2:** Morphological observation of the myocardial tissue of rats in the cardiac hypertrophy, low-dose tanshinone IIA, high-dose tanshinone IIA and control groups (× 400) Note: **A**. the control group; **B**. the cardiac hypertrophy group; **C**. the low-dose tanshinone IIA group; **D**. the high-dose tanshinone IIA group.

### Effect of tanshinone IIA on the serum cTn-I, ADMA and NO levels of SHRs

The serum cTn-1, ADMA and NO levels of rats in the cardiac hypertrophy, low-dose tanshinone IIA, high-dose tanshinone IIA and control groups were detected by ELISA. The results (Table 2) showed that the serum cTn-I and ADMA levels was significantly elevated and the serum NO level was significantly reduced in the cardiac hypertrophy group when compared with the control group (all *P* < 0.05). While compared with the cardiac hypertrophy group, the serum cTn-I and ADMA levels in the low- and high-dose tanshinone IIA groups decreased significantly, but the serum NO level increased significantly (all *P* < 0.05). No significant difference was found in serum cTn-I, ADMA and NO levels between the low- and high-dose tanshinone IIA groups (all *P* > 0.05).

**Table 2:** The effect of tanshinone IIA on the serum cTn-I, ADMA and NO levels

Group	cTn-I (pg/mL)	ADMA (ng/mL)	NO (pg/mL)
Control group	31.24 ± 3.71	1.13 ± 0.34	23.30 ± 5.51
Cardiac hypertrophy group	43.82 ± 4.44*	6.09 ± 2.17*	9.84 ± 2.73*
Low-dose tanshinone IIA group	33.39 ± 4.03^#^	1.26 ± 0.93^#^	20.61 ± 4.38^#^
High-dose tanshinone IIA group	33.87 ± 4.11^#^	1.21 ± 0.65^#^	18.77 ± 4.90^#^

Note: cTn-I, cardiac troponin I; ADMA, asymmetric dimethylarginine; NO, nitric oxide; *, *P* < 0.05 compared with the control group; ^#^, *P* < 0.05 compared with the cardiac hypertrophy group.

### Comparison of the mRNA expressions of COL1A1 and COL3A1 in the myocardial tissue among the four groups

The mRNA expressions of COL1A1 and COL3A1 in the myocardial tissue of rats in the cardiac hypertrophy, low-dose tanshinone IIA, high-dose tanshinone IIA and control groups were detected by qRT-PCR. As Figure 3 displays, the mRNA expressions of COL1A1 and COL3A1 increased significantly in the cardiac hypertrophy group when compared with the control group (all *P* < 0.05). Compared with the cardiac hypertrophy group, the mRNA expressions of COL1A1 and COL3A1 decreased significantly in the low- and high-dose tanshinone IIA groups (all *P* < 0.05). No significant difference was found in the COL1A1 and COL3A1 mRNA expressions among the control, low-dose tanshinone IIA and high-dose tanshinone IIA groups (all *P* > 0.05).

**Figure 3:** The mRNA expression changes of COL1A1 and COL3A1 in the myocardial tissue of rats in the cardiac hypertrophy, low-dose tanshinone IIA, high-dose tanshinone IIA and control groups Note: *, *P* < 0.05 compared with the control group; ^#^, *P* < 0.05 compared with the cardiac hypertrophy group.

### Effect of tanshinone IIA on the Cys-C/Wnt signaling pathway-related protein expressions in the myocardial tissue of SHRs

Western blotting results (Figure 4) showed that the expressions of Cys-C, Wnt2, β-catenin and WISP-1 in the myocardial tissue of rats in the cardiac hypertrophy group were significantly higher than those in the control group (all *P* < 0.05). Compared with the cardiac hypertrophy group, the expressions of Cys-C, Wnt2, β-catenin and WISP-1 significantly decreased in the low- and high-dose tanshinone IIA groups (both *P* < 0.05). Besides, no significant difference was found in Cys-C, Wnt2, β-catenin and WISP-1 expressions among the control group, the low-dose tanshinone IIA group and the high-dose tanshinone IIA group (all *P* > 0.05). These results indicated that tanshinone IIA might protect rats from cardiac hypertrophy through inhibiting the Cys-C/Wnt signaling pathway.

**Figure 4:** The expressions of the Cys-C/Wnt signaling pathway-related proteins in the myocardial tissue of rats in the cardiac hypertrophy, low-dose tanshinone IIA, high-dose tanshinone IIA and control groups Note: **A**. Western blotting analysis of Cys-C, Wnt2, β-catenin and WISP-1 expressions in the four groups; **B**. the histogram of Cys-C, Wnt2, β-catenin and WISP-1 expressions in the four groups; *, *P* < 0.05 compared with the control group; ^#^, *P* < 0.05 compared with the cardiac hypertrophy group; WISP-1, Wnt1-inducible signaling pathway protein-1.

### Comparison of eNOS expression and p-eNOS (Ser1177) phosphorylation level in the myocardial tissue among the four groups

The eNOS and p-eNOS expressions in the myocardial tissue of rats in the cardiac hypertrophy, low-dose tanshinone IIA, high-dose tanshinone IIA and control groups were detected by Western blotting. The results (Figure 5) revealed that the eNOS and p-eNOS (Ser1177) expressions in the cardiac hypertrophy group were significantly lower than those in the control group, but the Nox4 expression was significantly higher (all *P* < 0.05). Compared with the cardiac hypertrophy group, the eNOS and p-eNOS (Ser1177) expressions were elevated significantly in the low- and high-dose tanshinone IIA groups, but the Nox4 expression was significantly reduced (all *P* < 0.05). No significant difference was found in eNOS and p-eNOS (Ser1177) expressions between the low- and high-dose tanshinone IIA groups (*P* > 0.05). The eNOS expression in the cardiac hypertrophy group was inhibited, but tanshinone IIA can significantly improve the phosphorylation of p-eNOS (Ser1177) in the myocardial tissue of rats to enhance the activity of eNOS and can also down-regulate the Nox4 expression to reduce the vitality of NADPH, which ultimately protects against cardiac hypertrophy in SHRs.

**Figure 5:** The expressions of eNOS and p-eNOS (Ser1177) in the myocardial tissue of the rats in the cardiac hypertrophy, low-dose tanshinone IIA, high-dose tanshinone IIA and control groups Note: **A**. Western blotting analysis of eNOS and p-eNOS (Ser1177) expressions in the four groups; **B**. the histogram of eNOS and p-eNOS (Ser1177) expressions in four groups; *, *P* < 0.05 compared with the control group; ^#^, *P* < 0.05compared with the cardiac hypertrophy group; eNOS, endothelial NO synthase; p-eNOS, phosphorylated eNOS.

## DISCUSSION

Our study aimed to investigate the protective effect of tanshinone IIA against cardiac hypertrophy in SHRs through the Cys-C/Wnt signaling pathway. We found that tanshinone IIA can inhibit cardiac hypertrophy in SHRs through inhibiting the Cys-C/Wnt signaling pathway.

Cardiac hypertrophy is an adaptive response to stress or injury and can induce diverse signaling pathways, thereby leading to the activation of transcription factors and the reprogramming of gene expressions [18]. It is featured by increased size of cells, elevated synthesis of proteins, as well as heightened organization of sarcomeres [19]. Tanshinone IIA, a famous Chinese drug, can ameliorate angiotensin II-induced cardiomyocyte hypertrophy by inhibiting its downstream factors c-fos and c-jun mRNA expressions and reducing protein synthesis rate of cardiomyocytes [20], which is in consistent with our findings that compared with the cardiac hypertrophy group, groups treat with tanshinone IIA had decreased swelling degree of myocardial cells and area of single myocardial cell.

Our study found that rats in the cardiac hypertrophy group had obviously increased serum cTn-I level, and COL1A1 and COL3A1 mRNA expressions than the control group. cTn-I is a marker of cardiac hypertrophy with good specificity and sensitivity, and it is significantly increased after myocardial injury [21]. Accumulation of collagens (COL1A1 and COL3A1) is the main cause of cardiac fibrosis featured by the excessive accumulation of the extracellular matrix (ECM) [22, 23]. Cardiac fibrosis plays a very important role in the pathogenesis of cardiac hypertrophy [24]. Compared with the cardiac hypertrophy group, the serum cTn-I level and the mRNA expressions of COL1A1 and COL3A1 were significantly decreased in both the low-dose and high-dose tanshinone IIA groups, and no significant difference was found between the low-dose and high-dose tanshinone IIA groups, suggesting that tanshinone IIA has a protective effect on cardiac hypertrophy.

Through the Western blotting analysis, we found that the eNOS and p-eNOS (Ser1177) expressions in the cardiac hypertrophy group were significantly lower than those in the control group, but tanshinone IIA can significantly up-regulate the phosphorylation level of p-eNOS (Ser1177) in myocardia to enhance the activity of eNOS. eNOS plays an important role in cardiovascular system and in the regulation of cell apoptosis, cell growth, protein synthesis and metabolism, and it is also an important signal molecule involved in the production of endogenous NO [25, 26]. The phosphorylation of p-eNOS (Ser1177) can enhance the activity of eNOS [27]. Tanshinone IIA can protect the heart through promoting the phosphorylation of eNOS and stimulating the eNOS mRNA expression in myocardium [28, 29].

Besides, compared with the control group, the serum ADMA level in the cardiac hypertrophy group was significantly increased and the serum NO level was significantly decreased, respectively. However, the serum ADMA level was decreased and the serum NO level was increased after treated by tanshinone IIA. NO, which is produced by a family of enzymes called nitric oxide synthases, plays a key role in the state of blood vessel tone and hence blood pressure regulation [30]. The increase of ADMA can result in the reduction of NO by disrupting the synthesis of NO, which can lead to a variety of cardiovascular diseases and induce cardiac hypertrophy and interstitial fibrosis [31, 32]. Tanshinone IIA gives rise to arteriolar vasodilation caused by increased production of NO and lower BP [33].

Furthermore, we also found that the Cys-C and Wnt expressions in the myocardial tissue of rats in the cardiac hypertrophy group were significantly higher than those in the control group, indicating that Cys-C and Wnt expressions is positively related to cardiac hypertrophy. A previous study demonstrated that the elevation of Cys-C can evoke an inhibition of cathepsin B, and an accumulation of collagen I, collagen III and fibronectin in the ischaemic area of the myocardium, indicating a stimulatory role of Cys-C in cardiac hypertrophy [34]. Additionally, the activation of Wnt signaling pathway is responsible for the growth of hypertrophy [8, 35, 36]. After treated by tanshinone IIA, the Cys-C and Wnt expressions decreased significantly, suggesting that tanshinone IIA may have a protective effect on cardiac hypertrophy in SHRs through the inhibition of the Cys-C/Wnt signaling pathway.

In summary, the present study mainly clarified that tanshinone IIA can protect against cardiac hypertrophy in SHRs through suppressing the Cys-C/Wnt signaling pathway, which yields a new understanding of the therapeutic effect of tanshinone IIA on cardiac hypertrophy. However, due to time constraint, we did not analyze the association between the protective effect of tanshinone IIA with different concentrations and the degree of cardiac hypertrophy improvement. Therefore, further experiments are needed to investigate whether the protective effect of tanshinone IIA against cardiac hypertrophy differs with their concentrations, so as to lay a solid foundation for the clinical application of tanshinone IIA.

## MATERIALS AND METHODS

### Ethics statement

All animal experiments were conducted in strict accordance with the national animal experimental requirements and were approved by the Animal Ethics Committee (AEC) of Tongji Hospital, Huazhong University of Science and Technology. All efforts were made to minimize suffering.

### Animal grouping and drug administration

Experiments were performed on male SHRs and Wistar-Kyoto (WKY) rats (clean animals), aging 17 weeks and weighting 256.63 ± 29.47 g, and they were all purchased from Institute of Zoology, Chinese Academy of Sciences (Shanghai, China). Before experiment, all experimental rats had normal feed and consumption of water, and were raised at 25 ± 1°C with 50% humidity for 4 weeks. Subsequently, 30 SHRs were randomly divided into three groups: the cardiac hypertrophy group (S17), the low-dose tanshinone IIA group (S17) and the high-dose tanshinone IIA group (S17), with 10 rats in each group. Besides, 10 WKY rats (W17) were set as the control group. Rats in the low-dose tanshinone IIA group were given 1 mg/kg tanshinone IIA (Nou xin kang®, The First Biochemical Pharmaceutical Co. Ltd, Shanghai, China) through intraperitoneal injection from the first day of experiment, while rats in the high-dose tanshinone IIA group were given 10 mg/kg tanshinone IIA through intraperitoneal injection once a week [37]. Rats in the cardiac hypertrophy and control groups were intraperitoneally injected with 1 ml sterile water once a day. After 4 weeks of culture, the rats in the four groups were executed under anesthesia to obtain myocardial tissue and serum which were then stored at -80°C for further experiment.

### Determination of blood pressure (BP) in rat tail artery

The treated rats were maintained under the condition of 37°C for 15 min to make the blood vessels in the rat tail fully expanded. Subsequently, the rats were carefully loaded into a fixed set with fixed net, and an appropriate tail sleeve was used to sleeve the proximal part of rat tail root. After fixation, the rats were covered with the lid. The whole process was completed very quickly and softly. The BP in rat tail artery was measured when the rats were in a stable condition. An indirect method was used to measure the systolic arterial pressure (SAP) of all rats. The measurement was repeated for 5 times, and the mean systolic blood pressure (SBP) of each rat was calculated. All operations were performed in conscious rats, and SBP > 20 kPa (150 mmHg) was regarded as hypertension [38].

### Measurement of myocardial weight indexes

After the last injection of tanshinone IIA, all rats were fasted for 12 h but had free access to water, and then their body weights (BWs) were measured. The heart of each rat was taken out with the thoracic cavity opened, was washed with pre-cooled physiological saline and then was dried with filter paper for determining the heart weight (HW) and the left ventricular weight (LVW). Subsequently, the HW/BW and LVW/BW were calculated.

### Morphological observation of left ventricular myocardium

The left ventricular tissue samples were extracted and fixed in 4% paraformaldehyde, followed by phosphate buffer saline (PBS) wash, gradient ethanol dehydration and xylene transparency. After that, xylene was diluted by distilled water, and the samples were waxed in paraffin melted in the constant temperature chamber and then were transferred into an embedding device containing melted paraffin. When the liquid paraffin became solid after cooling, the paraffin-embedded tissue samples were fixed in object sland and sliced by paraffin slicing machine, followed by dewaxing in ethanol for the preparation of tissue sections. Next, the sections were dyed by hematoxylin-eosin (HE) for 5 min. After washing, the sections were treated with 0.5% alcohol solution of eosin for 2 min for coloration, followed by ethanol dehydration, xylene transparency and neutral gum sealing. The sections were observed under Nikon ECLIPSE 80i biological microscope (Nikon Corp., Tokyo, Japan), and 5 fields of vision were randomly selected for photographing. Automatic morphology measuring instrument (HPIAS21000, China) was used to measure the diameter and area of myocardial cells in the left ventricle, with each films measured for 6 times to obtain the average value.

### Quantitative real-time polymerase chain reaction (qRT-PCR)

The total RNA of the myocardial tissue was extracted using PCR kit (Vazyme Biotech Co., Ltd, Nanjing, China), and was reversely transcribed using Reverse Transcription kit (Promega, Madison, WI, USA) to synthesize cDNA. The mRNA expressions of COL1A1 and COL3A1 were detected by qRT-PCR. Glyceraldehyde-3-phosphate dehydrogenase (GAPDH) was regarded as the internal reference, and the primers were designed and synthesized by Shanghai Sangon Biotechnology Co., Ltd. (Shanghai, China) using real-time PCR machine (Eppendorf, Hamburg, Germany) (Table 3). The PCR reaction system was as follows: 10 μl of SYBR Green Master (Rox) (Roche, Basel, Switzerland), 1 μl of forward primer, 1 μl of reverse primer, 1 μl of cDNA and 7 μl of diethylpyrocarbonate (DEPC), totally 20 μl. The standard process of PCR amplification reaction was: pre-denaturation at 95°C for 5 s, and 40 cycles of 95°C for 5 s, 60°C for 31 s and 95°C for 20 s. Ct was used for result analysis, and the relative expressions of COL1A1 and COL3A1 were calculated.

**Table 3:** The primer sequences of COL1A1, COL3A1 and GAPDH for qRT-PCR

Gene	Primer sequence (5′-3′)
COL1A1	F: TCAAGATGGTGGCCGTTACT
	R: CATCTTGAGGTCACGGCATG
COL3A1	F: TGGGATGCAACTACCTTGGT
	R: AGGTGTAGAAGGCTGTGGAC
GAPDH	F: GTGACAGCCGCATCTTCTTG
	R: TGACTGTGCCGTTGAACTTG

Note: qRT-PCR, quantitative real-time polymerase chain reaction; GAPDH, glyceraldehyde-3- phosphate dehydrogenase; F, forward; R, reverse.

### Enzyme linked immunosorbent assay (ELISA)

The experiment was conducted according to the instructions of cardiac troponin I (cTn-I) (Life Diagnostics, West Chester, PA, USA), asymmetric dimethylarginine (ADMA) (R&D Systems, Minneapolis, MN, USA) and nitric oxide (NO) (NeoScientific, Cambridge, MA, USA) ELISA kits. Serum samples of rats were added into a 96-well plate at the bottom of which the serum combined with the capture antibody, and then was incubated at room temperature for 1 h. After fully washing, the enzyme-labeled antibody was added, followed by incubation for 30 min. Next, the plate was washed 3 times, and the chromogenic substrate tetramethylbenzidine (TMB) was added. The reaction was terminated by adding sulphuric acid. The 96-well plate was read at 490 nM of the microplate reader, and the concentrations of cTn-I, ADMA and NO in samples were calculated based on the optical density (OD).

### Western blotting

The myocardial tissues of all rats were pounded by homogenizer and centrifuged at 4°C for 10 min at 12,000 r/min. Next, the supernatant was collected, and the bicinchoninic acid (BCA) kit was used to detect the protein concentration. A total of 60 μg total protein was separated by gel electrophoresis at 70 V for 120 min, transferred into polyvinylidene fluoride (PVDF) membrane, and then blocked by 5% bovine serum albumin (BSA) at room temperature for 1.5 h. The primary antibodies, including Cys-C (1 : 3000, ab109508), Wnt2 (1 : 3000, ab109222), β-catenin (1 : 5000, ab32572), Wnt1-inducible signaling pathway protein-1 (WISP-1) (1 : 1000, SC25441), nicotinamide adenine dinucleotide phosphate (NAPDH) oxidase 4 (Nox4) (1 : 1000, ab133303), endothelial NO synthase (eNOS) (1 : 3000, ab66127) and phosphorylated eNOS (p-eNOS) (Ser1177) (1 : 2500, ab75639), were incubated at room temperature for 2 h and then maintained at 4°C overnight. All antibodies were purchased from Abcam Company (Cambridge, MA, USA) and Santa Cruz Biotechnology (Santa Cruz, California, USA). The membrane was washed by Tris-buffered saline-Tween (TBST) 3 times, and the goat anti-rabbit IgG labeled with horseradish peroxidase (HRP) was added (1 : 5000) for incubation at room temperature for 1.5 h. The protein bands were developed after dyeing by enhanced chemiluminescence (ECL) reagents. Image software was applied to analyze the gray level of protein expression. β-actin was regarded as the internal reference, and the ratio of target protein to the density of β-actin was regarded as the relative expression of target protein.

### Statistical analysis

SPSS 19.0 statistical software (SPSS Inc., Chicago, IL, USA) was used for data analysis. Measurement data were expressed as mean ± standard deviation (SD). The one-way analysis of variance (ANOVA) was used to compare multiple groups, and the least square difference method (LSD) was applied to compare two groups. *P* < 0.05 was considered statistically significant.
